# MicroRNA-8126-Mediated Antioxidant Stress Attenuates Isoflurane-Induced Hippocampal Neurotoxicity in Developing Rats

This article has been retracted.

**DOI:** 10.1155/2022/1618577

**Published:** 2022-08-17

**Authors:** Wen Pan, WenFeng Xiao, LingShuai Xue, Chao You

**Affiliations:** ^1^Department of Neurosurgery, West China Hospital, Sichuan University, Chengdu 610044, China; ^2^Department of Neurosurgery, Sichuan Mianyang 404 Hospital, Mianyang 621053, Sichuan, China; ^3^Department of Neurosurgery, Shougang Shuigang Hospital, Beijing 100043, China

## Abstract

**Objective:**

To investigate the effect of microRNA-8126 (*miR-8126*) on isoflurane-induced hippocampal neurotoxicity in rats.

**Methods:**

A rat isoflurane nerve injury model was constructed. The expression of *miR-8126* in the hippocampal region of normal and injured rats was measured by qRT-PCR; synaptic density protein-95, PAK-3 (p21-activated kinase-3) and apoptosis-related proteins cytochrome C, cleaved caspase-3, and cleaved PARP were detected by Western blot. The Cytochrome C, cleaved-caspase-3, and cleaved PARP expression was detected by WB, as well as GSH-Px, CAT, SOD, and ROS.

**Results:**

*miR-8126 was* lowly expressed in the isoflurane-treated rat hippocampal region and in rat hippocampal neuronal cells, and the expression of apoptosis-related proteins and apoptosis levels were significantly increased, and neural activity, cell activity, and proliferation capacity were significantly decreased. Oxidative stress levels and ROS content were significantly increased; overexpression of *miR-8126* in the rat hippocampal region significantly inhibited oxidative stress and apoptosis. Overexpression of *miR-8126* in rat hippocampal neural progenitor cells significantly increased cell activity, proliferative capacity, and significantly smaller mitochondrial size and it decreased ROS content and oxidative stress levels and apoptosis-related protein expression compared to isoflurane-treated cells; while inhibition of *miR-8126* expression in rat hippocampal neuronal cells significantly decreased cell activity, proliferative capacity, and mitochondrial size compared to the control group. In contrast, inhibition of miR-8126 expression in rat hippocampal neuronal cells resulted in a further decrease in cell activity, proliferation capacity, and significantly larger mitochondrial size and increased expression of apoptosis-related proteins compared with the control group. *miR-8126* regulates the activity of rat hippocampal neuronal cells by targeting ATF4.

**Conclusions:**

*miR-8126* attenuates isoflurane-induced hippocampal neurotoxicity in rats by mediating antioxidative stress.

## 1. Introduction

Sevoflurane, the most commonly used inhalation anesthetic in pediatric anesthesia, has become an essential tool for anesthesiologists because of its low airway irritation, rapid induction, and quick awakening. However, questions about its safety have also arisen. So, do general anesthetic drugs affect the development of the central nervous system of the child or not? A growing number of studies have shown that general anesthetic drugs can cause neurodevelopmental damage in nematodes, zebrafish, rats, guinea pigs, pigs, and macaques. The results of these animal studies are gradually being corroborated by clinical evidence. Several retrospective studies have confirmed that general anesthesia can indeed cause developmental brain damage, such as learning disabilities. Researchers at the Mayo Clinic studied the academic performance and medical records of 5,357 young children in a Minnesota community and found that children who received two surgeries and anesthesia before the age of 3 were at a 59% increased risk of experiencing learning impairment [1]. The risk of learning impairment was 2.6 times higher for children with 3 or more surgical anesthetics than for children of the same age group. Of particular note, children who received multiple anesthesia exposures before the age of 4 had cognitive scores that were 2 times lower than the normal predictive value, consistent with results shown in another study of a large population of 228,961 children [1]. In addition, the longer a child is anesthetized, the greater the risk of developing impaired learning function. Another case report showed varying degrees of neurodevelopmental delay in three infants within 2 months of age who received general anesthesia, and a brain magnetic resonance scan᧿ at 2–3 years of age showed abnormal bilateral cortical and subcortical symmetrical changes [2]. In fact, in terms of mechanistic studies, there has been a greater shift towards animal experiments. There is growing evidence that the most commonly used clinical inhalation anesthetics cause abnormal neurobehavioral alterations [3]. Studies from rodents and nonhuman primates have shown that early sevoflurane exposure leads to decreased learning memory, increased anxiety-like behavior, and social impairment in adulthood, and that the molecular mechanisms responsible for these alterations involve multiple components of neuronal proliferation, differentiation, autophagy, oxidative stress, apoptosis, and synaptic development.

MicroRNAs are a class of small molecular single-stranded noncoding small RNAs that have been highly conserved over the course of biological evolution and are involved in a variety of biological processes, including apoptosis, cancer development, and cell development, such as bone and muscle development [3]. Recent studies have revealed that METH can induce microRNA expression and then regulate the expression of related genes in a post-transcriptional manner, which in turn activates associated intracellular signaling pathways causing neuronal toxic damage (iv). In 2012, German scientists found that miR-181a overexpression reduced GluA2 receptor expression and downregulated the frequency of microexcitatory postsynaptic currents (mEPSC), demonstrating that METH can alter miR-181a expression to regulate neurosynaptic plasticity [4]. These comprehensive analyses aimed to reveal the underlying molecular regulatory mechanisms of miR-8126 on isoflurane-induced hippocampal neurotoxicity.

## 2. Materials and Methods

### 2.1. Establishment of an Isoflurane Hippocampal Nerve Injury Model in Rats

Forty 7-day-old SD (Sprague–Dawley) rats were purchased from the Experimental Animal Centre of Tongji Medical College, Huazhong University of Science and Technology (Wuhan, China). The rats were then numbered according to their body weight and randomly divided into two groups: the isoflurane-treated group (30 rats) and the control group (10 rats). Rats in the isoflurane-treated group were incubated in 1.8% isoflurane, 21% oxygen and nitrogen, and rats in the control group were incubated in 21% oxygen, and 78% nitrogen for 12 h. Rats were then executed, and tissues from the hippocampal region were extracted for subsequent experiments.

### 2.2. Rat Lateral Brain Injection

Thirty rats were randomly divided into three groups of 10 rats each, numbered according to their body weight. The rats were injected by lateral brain injection, with the injection points located relative to bregma: anterior-posterior, −2.5 mm; lateral, ±2.7 mm; dorsal, 2.9 mm; saline, miR-negative control; and miR-8126 mimics (purchased from RiboBio (Shanghai, China)) were injected intracranially into the rats of each group, which were categorised as blank group, miR-NC group, and miR-NC group. The miR-NC group and miR-8126 group were recorded as blank groups, miR-NC group, and miR-8126 group. After 12 h of injection, the rats were placed in a room containing 1.8% isoflurane and 21% oxygen and nitrogen for 12 h. The rats were then executed and tissues from the hippocampus were extracted for subsequent experiments: five rats from each group were used for tissue sectioning; the other five rats were used for qRT-PCR, western blot, and oxidative stress assay.

### 2.3. qRT-PCR and WB

The qRT-PCR and WB assays were performed to detect mRNA and protein expression levels of genes.

In brief, total RNA was isolated using the TRIzol kit (Thermo Fisher Scientific). RNA samples were reverse transcribed using the PrimeScript® miRNA cDNA synthesis kit (TaKaRa, Dalian, China) or the PrimeScript® RT kit (TaKaRa). Real-time qPCR was performed on a 7500 real-time PCR system (Applied Biosystems, CA, USA) using SYBR green qPCR master mix kit (Thermo Fisher Scientific). The relative expression of genes was examined using the 2−ΔΔCT method.

Total protein in cells was isolated using RIPA cell lysis buffer. After measuring the concentration using the BCA kit, protein samples were separated by SDS-PAGE and loaded onto PVDF membranes. After blocking in 5% skim milk for 1 h, the blotted bands were hybridized with primary antibody overnight at 4°C and with horseradish peroxidase-conjugated secondary antibody for 2 h at 37°C. The blotted bands were visualized with ECL reagent (Beyotime Biotechnology Co., Ltd., Shanghai, China) and analyzed by Image J (Bio-Rad, Hercules, CA, USA).

### 2.4. Oxidative Stress Assay

ROS in the tissues was measured by the MitoSOX kit (Invitrogen, Carlsbad, CA, USA) was used for ROS measurement.

### 2.5. TUNEL

The TUNEL assay was used to detect apoptosis in the rat hippocampus using the TUNEL kit (Roche, Basel, Switzerland). All procedures were carried out strictly according to the instructions. Condensed nuclei were TUNEL-positive cells, i.e., apoptotic neuronal cells. Five fields of view were randomly selected for observation and counting.

### 2.6. Mitochondrial Function Assay

Mitochondrial size was analyzed using the mitochondrial swelling assay, mitochondrial morphology was observed using transmission electron microscopy, and intracellular calcium concentration was analyzed using intracellular calcium presentation to confirm the integrity of mitochondrial function.

### 2.7. Immunofluorescence

Groups of cells grown on glass coverslips were rinsed, washed three times with PBS, and fixed in 4% paraformaldehyde for 15 min at 4°C. The cells were treated with 0.5% Triton-100× for 20 min. MAP-2 primary antibody was added and incubated overnight at 4°C. Cells were washed with PBS and incubated with fluorescent sheep anti-rabbit secondary antibody for 1 h at 37°C. Cells were observed first by fluorescence microscopy.

### 2.8. Cell Activity Assay

Activity of hippocampal neurons was detected by CCK-8 and EdU staining. The proportion of apoptotic cells was detected by flow cytometry using Annexin-V with PI labeling, and apoptotic morphological changes in the nucleus were observed using Hoechst 33258 staining.

### 2.9. Dual Luciferase Gene Reporter

The 3′-UTR binding sequence of miR-8126 to ATF4 was predicted by the line prediction software Target Scan (https://www.targetscan.org/vert_72/), and ATF4 wild-type WT and 3′-UTR binding sequences were synthesized by Biotech Bioengineering Ltd. (Shanghai, China), and inserted into pMIR-REPORTTM (Thermo Fisher Scientific, CA, USA) luciferase reporter vector. WT plasmid, MT plasmid, and miR-8126 mimics and miR negative control were cotransfected into 293T cells using the Lipofectamine 2000 transfection kit (Invitrogen, USA), and the cells were lysed after 8126h and transfected by a dual-luciferase reporter assay system (Promega Corporation, WI, USA) to detect the intensity of luciferase activity.

## 3. Results

### 3.1. miR-8126 is Lowly Expressed in the Hippocampal Region of Isoflurane-Treated Rats

12 hours of isoflurane, oxygen, and nitrogen were given to rats. 12 hours were spent incubating control rats in 21% oxygen and 78% nitrogen. After killing the rats, the hippocampi were removed for studies. Synaptic density protein-95 and PAK-3 were detected by qRT-PCR. The mRNA expression of PAK-3 was significantly decreased (*P* < 0.05) compared with the control group (Figure 1(a)), and the Western blot results were consistent (*P* < 0.05) (Figure 1(b)), indicating that the hippocampal activity of rats was reduced after isoflurane treatment; and cytochrome C, cleaved caspase-3, and cleaved PARP increased significantly (*P* < 0.05) (Figure 1(c)); TUNEL immunohistochemical staining was utilized for detection of neuron apoptosis, which indicated isoflurane's neurotoxicity. MiR-8126 was low in isoflurane-treated rats' hippocampus (*P* < 0.05) (Figure 1(e)).

### 3.2. Overexpression of miR-8126 in the Rat Hippocampus Effectively Inhibits Isoflurane-Induced Neurotoxicity

Using the lateral brain injection approach, we injected saline, miR-8126 mimics, and miR negative control into newborn rats' brains. After 12 h in oxygen containing 1.8% isoflurane and 21% oxygen and nitrogen, rats were executed and their hippocampi were taken for research. The PSD-95 and PAK-3 mRNA levels were significantly higher (*P* < 0.05) in the miR-8126 group compared to the blank and miR-NC groups (Figure 2(a)), and western blot showed similar results (P&T). Western blot showed lower expression of cytochrome C, cleaved caspase-3, and cleaved PARP in the hippocampus of miR-8126 rats (*P* < 0.05) (Figures 2(b) and 2(c)). MiR-8126 exhibited considerably fewer apoptotic cells than miR-NC (*P* < 0.05) (Figure 2(d)).

### 3.3. Overexpression of *miR-8126* Inhibits Oxidative Stress in the Hippocampal Region of Isoflurane-Treated Rats

In the hippocampus of isoflurane-treated rats, the activities of oxidative stress-related proteins SOD, GSH-Px, and catalase (CAT) were significantly lower and MDA levels were increased (*P* < 0.05) compared with the nonisoflurane-treated control group (Figure 3(a)). In contrast, overexpression of miR-8126 in the brain increased the enzymatic activities of SOD, GSH-Px, and CAT, while MDA isoflurane therapy-enhanced hippocampus neuronal oxidative damage (*P* < 0.05) (Figure 3(b)). The miR-8126 group's hippocampus had less oxidative damage than the miR-NC group (*P* < 0.05) (Figure 3(b)). MiR-8126 overexpression inhibits oxidative stress in isoflurane-treated rats' brains.

### 3.4. Overexpression of miR-8126 Enhances the Activity of Isoflurane-Treated Rat Hippocampal Neuronal Cells

The isolated cultured cells were rat hippocampus neuronal cells, according to NSE and MAP-2 labeling (Figure 4(a)). By qRT-PCR, isoflurane-treated cells had decreased miR-8126 expression than untreated cells (*P* < 0.05) (Figure 4(b)).

To create rat hippocampus neuronal cells that persistently overexpressed and inhibited miR-8126, we transfected miR-8126 mimics and inhibitors using the lipofectamine 2000 transfection kit (Invitrogen, USA). After 48 h of transfection, qRT-PCR detected a significant increase in miR-8126 expression in rat hippocampal neuronal cells in the miR-8126 group and a significant decrease in the miR-IN group (*P* < 0.05) (Figure 4(c)), indicating that overexpression or interference of miR 8126 in the rat hippocampal neuronal cell line was successfully constructed.

The qPCR assay of PSD-95 and PAK-3 mRNA levels showed that, compared with the miR-NC group, the miR-8126 group had considerably higher mRNA levels, whereas the miR-IN group had significantly lower mRNA levels (*P* < 0.05) (Figure 4(d)); Western blot results confirmed these results. The qRT-PCR results was consistent Western blot results (Figure 4(e)).

Intracellular Ca2+ imaging was used to measure the activity of rat hippocampus neuronal cells in each group. The miR-8126 group had a considerably higher inward flow of Ca2+ in the presence of KCl than the miR-NC group, whereas the miR-IN group had a significantly lower inward flow of Ca2+ (*P* < 0.05) (Figure 4(f)).

MTT assay for cell activity showed that miR-8126 group cells had considerably higher activity than miR-NC group cells at 8126 h, 48 h, and 72 h; miR-IN group cells had significantly lower activity than miR-NC group cells at 8126 h, 48 h, and 72 h (Figure 4(g)).

The EdU infiltration assay was used to detect cellular DNA replication, and the results showed that the EdU positive rate of the miR-8126 group was significantly higher than that of the miR-NC group; the EdU positive rate of the miR-IN group was significantly lower (*P* < 0.05) than that of the miR-NC group (Figure 4(h)).

### 3.5. Overexpression of miR-8126 Attenuates Isoflurane-Mediated Oxidative Stress in Rat Hippocampal Neuronal Cells

Oxidative stress-related enzyme activities decreased in the miR-8126 group, but increased in the miR-IN group (*P* < 0.05) compared to the miR-NC group (Figure 5(a)).

Transmission electron microscopy examined each group's mitochondrial morphology. The mitochondrial volume in the miR-8126 group was considerably smaller than that in the miR-NC group (*P* < 0.05) (Figure 5(b)); the opening of mitochondrial permeable pore (mPTP) was measured by measuring mitochondrial Ca2+ permeability. The permeability of mitochondria to Ca2+ was then used to assess mPTP opening. The miR-8126 group displayed stronger resistance to Ca-mediated rise in mitochondrial swelling and permeability than the miR-NC group, but in the miR-IN group, swelling and permeability rose significantly (*P* < 0.05) more than in the miR-NC group (Figure 5(c)).

### 3.6. Overexpression of miR-8126 Attenuates Isoflurane-Mediated Apoptosis in Rat Hippocampal Neuronal Cells

Flow cytometry was used to compare the apoptosis rates of rat hippocampal neuronal cells in each group. The miR-8126 group had a lower apoptosis rate than the miR-NC group, while the miR-IN group had a higher apoptosis rate (all *P* < 0.05) (Figure 6(a)), indicating that overexpressed miR-8126 could inhibit apoptosis. Hoechst 33258 staining paired with fluorescence microscopy revealed morphological changes in apoptotic cells. The miR-8126 group had fewer apoptotic cells than the miR-NC group, whereas the miR-IN group had more (*P* < 0.05) (Figure 6(b)). Western blot detected the expression of proapoptosis-related proteins: cytochrome C, cleaved caspase-3, and cleaved PARP, and the results showed that the protein levels of proapoptosis-related proteins in the miR-8126 group were significantly decreased compared with the miR-NC group (both *P* < 0.05) (Figure 6(c)).

### 3.7. miR-8126 Enhances Rat Hippocampal Neuronal Cell Activity by Targeting ATF4

According to Target Scan (https://www.targetscan.org/vert_72/), ATF4 binds to miR-8126 in the 3′-UTR (Figure 7(a)). The luciferase reporter gene experiment indicated no significant difference between MT + mimics and MT + NC; however, WT + mimics had considerably lower luciferase activity than WT + NC (*P*0.01) (Figure 7(b)).

qRT-PCR results showed no significant difference in the mRNA expression level of ATF4 in 239 T cells in the miR-NC group compared with the blank group, while in the miR-8126 group, the expression level of ATF4 was significantly decreased compared with the blank group, and in the miR-IN group, the expression level of ATF4 was significantly increased compared with the blank group (*P* < 0.05) (Figure 7(c)). miR-IN -enhanced ATF4 expression relative to the blank group (all *P* < 0.05) (Figure 7(c)); Western blot results were consistent (all *P* < 0.05) (Figure 7(d)). MiR-8126 increases cell activity by inhibiting ATF4 activity, according to the preceding data.

## 4. Discussion

The mechanism of action of sevoflurane, a widely used inhalation anesthetic, is thought to be mediated through GABA receptors [122]. Previous studies have found that oxidative stress [5], autophagy [6], and microRNAs (e.g., microRNA188 and microRNA96) [7] may be involved in the induction of apoptosis by sevoflurane, which may be partially responsible for cognitive dysfunction. Our data show that activated caspase3 is mainly expressed in nonneuronal cells after sevoflurane exposure. Although neuronal apoptosis was detected in the hippocampal granular layer, the number of neurons did not change in adulthood. This result may be due to the fact that although neurons undergo apoptosis in the presence of sevoflurane during development, new neurons are constantly being formed, and it is possible that this constant replenishment results in no significant change in the number of neurons in adulthood compared with that after developmental sevoflurane exposure. Neuronal density did not show significant abnormalities 3 months after anesthetic exposure [8]. It has also been shown that continuous isoflurane exposure can cause neuronal death but does not impair spatial memory [9], showing that neuronal apoptosis may not be the main cause of cognitive dysfunction. We have demonstrated in the phase 1 experiments that miR-8126 has a determined protective effect on sevoflurane-induced hippocampal neuronal injury by both increasing neuronal cell viability and reducing neuronal apoptosis. So what is the mechanism or pathway of the protective effect of mjR-8126 on sevoflurane-induced hippocampal neuronal injury? In order to explore the possible mechanism or pathway of action, we proposed a concept and demonstrated it through experiments. miRNAs exert their biological effects by regulating their target genes, so we first started to explore the mechanism of the protective effect by the possible target genes regulated by miR-8126. A total of 212 possible target genes were predicted using the online software TargetScan for miR-8126 possible regulatory target genes. Among these target genes, the target genes of our interest were selected and analyzed for their complementary sites of interaction with miR-8126. Among the possible target genes regulated by miR-8126, we found ATF4. ATF4 plays an important role in many biological responses, such as the secretion of neurotransmitters, regulation of transcription factors, and glycogen metabolism [10, 11]. Approximately 1% to 2% of the protein in the brain is calmodulin kinase II [12]. The neuronal excitotoxic effects induced by sevoflurane are mainly associated with sevoflurane-induced calcium inward flow in hippocampal neurons, which is related to calmodulin function [13, 14]. Besides, microRNA-24 alleviates isoflurane-induced neurotoxicity in the rat hippocampus via attenuation of oxidative stress [15]. We again analyzed the complementary binding site of miR-8126 to the target gene ATF4 3′-UTR by TargetScan and envisioned to validate ATF4 as a miR-8126-regulated target gene by luciferase reporter gene system. Next, we designed rescue experiments to further validate that miR-219 exerts its protective effect on glutamate-induced hippocampal neuronal injury by regulating the target gene CaMXIIY. First, we constructed a recombinant expression vector pcDNA3-1-ATF4 for the target gene ATF4, and then examined whether the recombinant expression vector could effectively promote the expression of ATF4 protein after transfection with hippocampal neurons using Western blot. The results showed that the expression of ATF4 protein in hippocampal neurons was significantly increased after transfection with the recombinant expression vector pcDNA3-1-ATF4. Then, ATF4 was overexpressed in hippocampal neurons, and the cell viability of hippocampal neurons was examined again using an MTT assay to explore whether overexpression of CaMXIh could reverse the protective effect of overexpression of miR-219. The results showed that overexpression of ATF4 exacerbated the glutamate-induced decrease in neuronal cell viability and reversed the protective effect of miR-219 overexpression on hippocampal neurons. Through this rescue experiment, we further demonstrated that miR-219 exerts a protective effect on hippocampal neurons with glutamate-induced injury by regulating the expression of ATF4. In summary, this phase of study explored the possible mechanisms and signaling pathways by which miR-219 overexpression increased hippocampal neuronal cell viability and reduced neuronal apoptosis after glutamate-induced injury.

## 5. Conclusion

This study demonstrated that miR-219 could exert neuroprotective effects against glutamate-induced neuronal injury in the hippocampus by regulating the expression of the target gene ATF4 protein, inhibiting caspase-3 activity and increasing the Bcl-2/BaX ratio, and the P13 K/Akt cell signaling pathway was the signaling pathway for its protective effects. miR-219 had a positive protective effect against glutamate-induced neuronal cells. The positive protective effect of miR-219 against glutamate-induced excitotoxicity may be useful for further exploration of the mechanisms underlying the development of sepsis-associated encephalopathy in the future.

## Figures and Tables

**Figure 1:** Relative PSD-95 and PAK-3 mRNA level (a) and protein level (b) of hippocampus in isoflurane-treated rat or not; apoptosis-related protein expression level (c). TUNEL immunohistochemistry staining of rat hippocampus (d); relative *miR-8126* expression of hippocampus in isoflurane-treated rat or not (e); all ^*∗*^*P* < 0.05 and ^*∗∗*^*P* < 0.01* vs*. control, *N* = 5.

**Figure 2:** miR-8126 prohibits neurotoxicity induced by isoflurane in rat hippocampus. Relative PSD-95 and PAK-3 mRNA level (a) and protein level (b) of hippocampus in isoflurane-treated rat; apoptosis-related protein expression level (c) TUNEL immunohistochemistry staining of rat hippocampus; (d) all ^*∗*^*P* < 0.05, ^*∗∗*^*P* < 0.01* vs*. control, *N* = 5.

**Figure 3:** Overexpressed miR-8126 attenuates oxidative stress induced by isoflurane. Comparison of SOD, GSH-Px, CAT activity, and MDA content (a). MitoSOX staining for ROS in hippocampus (b). ^*∗*^*P* < 0.05 and ^*∗∗*^*P* < 0.01* vs*. control, ^#^*P* < 0.05 and ^*##*^*P* < 0.01* vs*. *miR-NC*. *N* = 5.

**Figure 4:** Overexpressed miR-8126 enhances isoflurane-treated hippocampal neurons viability. nSE ihc staining and MAP-2 immunofluorescent indicates hippocampal neurons phenotype (a); relative *miR-8126* expression of, in isoflurane-treated rat or not, hippocampal neurons (b); relative *miR-8126* expression after transfection (c); PSD- 95 and PAK-3 mRNA level (d) and protein level (e); intracellular Ca2+ levels were measured in fura-2-loaded hippocampal neurons (f); relative cell viability measured by CCK-8 kit (g) and EdU staining (h). All ^*∗*^*P* < 0.05 and ^*∗∗*^*P* < 0.01* vs*. *miR-NC*, *N* = 3. Neuron specific enolase, NSE; microtubule associated protein-2, MAP-2.

**Figure 5:** Overexpressed miR-8126 attenuates oxidative stress in isoflurane-treated hippocampal neurons. Comparison of SOD, GSH-Px, CAT activity, and MDA content (a). Mitochondrial appearance and size measured by TEM (b). Mitochondrial swelling level is detected relative percent of the initial OD at an absorbance of 540 nm (c). ROS assay using CM-H_2_ DCFDA (d). Imaging using a peroxide-selective probe H_2_-DCFDA (e). All ^*∗*^*P* < 0.05 and ^*∗∗*^*P* < 0.01* vs*. *miR-NC*, *N* = 3.

**Figure 6:** Overexpressed miR-8126 attenuates isoflurane-treated rat hippocampal neurons. Apoptosis ratio measured by flow cytometry (a); hoechst 33528 staining indicates apoptosis neurons (b); apoptosis-related proteins were detected by western blot (c). All ^*∗*^*P* < 0.05 and ^*∗∗*^*P* < 0.01* vs*. *miR-NC*, *N* = 3.

**Figure 7:** miR-8126 promotes rat hippocampal neuron viability by targeting ATF4. Target scan predicts *miR-8126* and ATF4 binding sequence (a); *miR-8126* binds to ATF4 mRNA and inhibits its activity by dual luciferase report assay (b); qRT-PCR (c); and Western blot (d). All ^*∗*^*P* < 0.05 and ^*∗∗*^*P* < 0.01.

## Data Availability

The data used to support the findings of this study are available from the corresponding author upon request.

## Additional Points

(1) *miR-8126* is hypoexpressed in the hippocampal region of isoflurane-treated rats. (2) *miR-8126* inhibits isoflurane-mediated neurotoxicity in the hippocampal region of rats. (3) Overexpression of *miR-8126* enhances the activity of isoflurane-treated rat hippocampal neuronal cells. (4) Overexpression of *miR-8126* attenuates isoflurane-induced oxidative stress damage in rat hippocampal neuronal cells. (5) *miR-8126* attenuates isoflurane-induced hippocampal neurotoxicity in developing rats through targeted inhibition of ATF4 activity.
